This article has been retracted.

# Downregulation of long non-coding RNA ANRIL suppresses lymphangiogenesis and lymphatic metastasis in colorectal cancer

**DOI:** 10.18632/oncotarget.9868

**Published:** 2016-06-07

**Authors:** Zhenqiang Sun, Chunlin Ou, Weiguo Ren, Xiang Xie, Xiayu Li, Guiyuan Li

**Affiliations:** ^1^ Key Laboratory of Carcinogenesis of Ministry of Health and Key Laboratory of Carcinogenesis and Cancer Invasion of Ministry of Education, Cancer Research Institute, Central South University, Changsha, 410000, Hunan, China; ^2^ Department of Gastrointestinal Surgery, Affiliated Tumor Hospital, Xinjiang Medical University, Urumqi, 830011, Xinjiang, China; ^3^ Department of Gastroenterology, The Third Xiangya Hospital of Central South University, Changsha, 410000, Hunan, China; ^4^ Hunan Key Laboratory of Nonresolving Inflammation and Cancer and Disease Genome Research Center, The Third Xiangya Hospital, Central South University, Changsha, 410000, Hunan, China; ^5^ Hunan Provincial Tumor Hospital and the Affiliated Tumor Hospital of Xiangya Medical School, Central South University, Changsha, 410013, Hunan, China; ^6^ Department of Coronary Artery Disease, Heart Center, First Affiliated Hospital of Xinjiang Medical University, Urumqi, 830011, Xinjiang, China

**Keywords:** ANRIL, colorectal cancer, lymphangiogenesi, lymphatic metastasis, invasion

## Abstract

This study aimed to investigate the effect of ANRIL on the lymphangiogenesis and lymphatic metastasis in colorectal cancer. Using RT-PCT and Northern blot, we detected ANRIL expression in tissues (cancer vs. normal) and cell lines (HCoEpic, SW480, HT29, LoVo and HCT116), finding that ANRIL was overexpressed in colorectal cancer. By statistical analysis, increased ANRIL was found to be in close association with TNM staging, Duke staging and lymphatic metastasis and poor prognosis. We down-regulated the high ANRIL expression in LoVo and HCT116 with lentivirus transfection, and found that the activity of cell mobility and invasion was remarkably reduced. And also we also identified that ANRIL down-regulation could suppress in-vitro tube formation HLECs invasion. In addition, we built a mouse model of colorectal cancer. In the mouse model, we recorded, after ANRIL downregulation, decreased tumor growth rates and tumor size and reduced lymphatic metastasis rate and frequency of transferred lymph nodes, LMVD and expressions of VEFG-C, VEGFR-3 and LYVE-1. Based on these findings, we concluded that increased ANRIL is promoter in the development of colorectal cancer. Through down-regulation of the overexpressed ANRIL, lymphangiogenesis may be suppressed and therefore lymphatic metastasis may be inhibited. On this ground, we suggest that ANRIL may be a therapeutic target for colorectal cancer.

## INTRODUCTION

Colorectal cancer is the third most frequently-diagnosed malignancy worldwide [1]. Due to its recurrence and metastasis, colorectal cancer is a leading type of cancer death, killing 26,804 males and 24,979 females in 2011 alone [2, 3]. Cancer metastasis is a process during which cancer cells disseminate form the primary tumor to organs. To our knowledge, tumor-associated lymphangiogenesis acts as a promoter in lymphatic metastasis, aiding to promote cancer cell recruitment to lymph nodes [4]. Increasing evidence has shown that lymphangiogenesis facilitate lymphatic metastasis in the development of colorectal cancer [5, 6]. Unfortunately, the mechanism how lymphangiogenesis happens in colorectal cancer remains to be explored.

Antisense non-coding RNA in the INK4 locus (ANRIL), a natural antisense transcript gene, is transcribed in the antisense orientation of *INK4b-ARF-INK4a* gene cluster [7]. ANRIL can talk with polycomb repressive complex-1 (PRC1) and -2 (PRC2) to form heterochromatin surrounding INK4b-ARF-INK4a locus and therefore repress the expression of such tumor-suppressor genes as *p15^INK4b^* and *p16^INK4a^* [8]. Evidence has shown that ANRIL overexpression is a promoter in cell proliferation and a suppressor in cell apoptosis in cancer development [9, 10]. Several studies have reported that ANRIL silencing could activate *p15^INK4b^* and *p16^INK4^*^a^ expression, causing suppression of cell proliferation and cellular senescence [11, 12]. To our knowledge, silencing of *p16^INK4a^* can lead to progression and invasion of colorectal cancer and further result in poor prognosis [13, 14]. A meta-analysis demonstrated that silencing of *p16^INK4a^* by hypermethylation could predict lymphovascular invasion and lymph node metastasis in the progression of colorectal cancer [15]. Interestingly, increased expression of ANRIL also closely correlated with advanced lymph node metastasis and poor prognosis [16]. In this context, we hypothesize that ANRIL, a suppressor for INK4a and INK4b loci, may be involved in the lymph node metastasis in colorectal cancer. Though most studies suggest that increased ANRIL promote lymph node metastasis, the mechanism ANRIL relates to it remains unexplained [17, 18]. As suggested, lymphangiogenesis generates new lymphatic vessels from the pre-existing lymphatics and thus facilitates lymphatic metastasis [19]. For this reason, we believe that lymphangiogenesis may be a junction where ANRIL exerts its function on lymphatic metastasis.

With the above hypothesis and conjecture, we start the present study. In our study, we perform close observation on colorectal cancer development in patients and in cancer cells, and build a mouse model of colorectal cancer, aiming to investigate the association between long non-coding RNA ANRIL and lymphangiogenesis and lymphatic metastasis in the progression of colorectal cancer.

## RESULTS

### ANRIL expression in the colorectal cancer and its association to clinic-pathologic features

RT-qPCR revealed that surgical specimens presented significantly higher expression of ARIL mRNA than normal colorectal mucosae (1.68 ± 0.22 vs. 0.52 ± 0.11, *t* = 39.88, *P* < 0.01) (Figure 1). ANRIL expression was defined as high level when it was higher than the mean ANRIL expression and as low level otherwise. As shown in Table 1, ANRIL expression was closely associated with TNM staging, Duke staging and lymphatic metastasis (all *P* < 0.05) while had no association with age, gender, tumor location, tumor size, degree of differentiation, depth of invasion and distant metastasis (all *P* > 0.05).

**Figure 1:** Expressions of ANRIL mRNA detected in surgical specimens and normal colorectal mucosae **A.** a presentation of ANRIL mRNA expression detected by RT-qPCR, with 1,3, 5 and 7 illustrating ANRIL expression of surgical specimens while 2,4 and 6 as representatives of normal colorectal mucosae; **B.** Statistical comparisons of the ANRIL mRNA expressions in surgical specimens and normal colorectal mucosae detected by RT-qPCR. Note: ANRIL, antisense non-coding RNA in the INK4 locus; RT-qPCR, real-time fluorescent quantitative polymerase chain reaction; *** refers to *P* < 0.001.

**Table 1:** Associations between ABRIL expression and clinicopathologic features in colorectal cancer

	Number of cases	ANRIL expression		*P*
		High	Low	
Age				
≤ 50	47	37	10	
> 50	61	45	16	0.55
Gender				
Male	59	42	17	
Female	49	40	9	0.26
Tumor location				
Colon	61	50	11	
Rectum	47	32	15	0.09
Tumor size				
≤ 5cm	54	45	9	
> 5cm	54	37	17	0.07
Differentiation level				
Low	23	15	8	
Moderate + high	85	67	18	0.18
TNM staging				
Stage I + II	59	50	9	
Stage III + IV	49	32	17	0.02
Dukes staging				
Stage A + B	56	49	7	
Stage C + D	52	33	19	0.01
Invasion depth				
Presence of plasma membrane invasion	74	54	20	
Absence of plasma membrane invasion	34	28	6	0.34
Lymphatic metastasis				
No	50	29	21	
Yes	58	53	5	< 0.01
Distant metastasis				
Yes	20	10	10	
No	88	72	16	0.08

Note: ANRIL, antisense non-coding RNA in the INK4 locus; ANRIL expression higher than the mean expression level is defined as high and otherwise low.

### Association between ANRIL expression and prognosis of colorectal cancer

We recorded 102 follow-ups of patients with colorectal cancer. The length of our follow-ups varied from 5~60 months, with a median follow-up time of 22 months. During the follow-up, we lost 2 patients with high ANRIL expression and 1 patient with low ANRIL expression. Among patients with high ANRIL expression, 5-year survival rate was 2.60% (2/77), significantly lower than that of 12.00% (3/25) among patients with low ANRIL expression (χ^2^ = 23.094, *P* < 0.001). The analyses using Kaplan-Meier demonstrated that high ANRIL expression may lead to poor prognosis in colorectal cancer (Figure 2). The Cox regression model showed that high ANRIL expression and lymphatic metastasis were independent risk factors for prognosis in colorectal cancer (Table 2).

**Figure 2:** ANRIL expression negatively associates with 5-year survival rate of patients with colorectal cancer Note: ANRIL, antisense non-coding RNA in the INK4 locus.

**Table 2:** Cox proportional hazards regression model for screening the risk factors for prognosis of colorectal cancer

	B	SE	Wald	Sig.	Exp (B)	95% CI for Exp (B)	
						Lower	Upper
ANRIL expression	4.12	0.57	53.10	0.00	61.68	20.36	186.92
Age	0.19	0.23	0.66	0.42	1.21	0.77	1.91
Gender	0.00	0.23	0.00	0.99	0.10	0.63	1.58
Tumor location	0.76	0.58	1.71	0.19	0.47	0.15	1.46
Tumor size	0.17	0.23	0.58	0.46	0.84	0.54	1.32
Differentiation level	0.06	0.28	0.05	0.82	0.94	0.55	1.62
TNM staging	0.50	0.77	0.41	0.52	1.65	0.36	7.50
Dukes staging	1.43	1.07	1.78	0.18	4.16	0.51	33.63
In vasion depth	0.41	0.25	2.67	0.10	1.50	0.92	2.46
Lymphatic metastasis	1.27	0.47	7.50	0.01	3.57	1.43	8.92
Distant metastasis	0.29	0.31	0.86	0.36	0.75	0.40	1.39

Note: ANRIL, antisense non-coding RNA in the INK4 locus; B, regression coefficient; SE, Standard error of regression coefficient; Wald, test statistics; df, degree of freedom. Sig., significance; Exp (B). index of the regression coefficients; CI, confidence interval.

### Associations of ANRIL expression with lymphangiogenesis-related factors and LMVD in surgical specimens

As presented in Figure 3A-3C, VEGF-C, VEGFR-3 and LYVE-1 concentrated in cytoplasm of cancer cell and mesenchymal cell, in form of granules colored as light to brownish yellow and in focal and diffused distribution. However, no obvious staining was observed in the cytomembrane and nucleus and no expression of VEGF-C, VEGFR-3 and LYVE-1 was found in the normal colorectal mucosae. In the surgical specimen, positive rates of VEGF-C, VEGFR-3 and LYVE-1 were 84.26% (91/108), 57.41% (62/108) and 39.81% (43/108), respectively. Positive expressions of VEGF-C, VEGFR-3 and LYVE-1 were significantly higher in the surgical specimens with high ANRIL expression compared with those with low ANRIL expression (all *P* < 0.05). Spearman correlation analysis revealed that ANRIL expression was in positive correlation with expressions of VEGF-C, VEGFR-3 and LYVE-1 (all *P* < 0.05) (Table 3). As shown in Figure 3D, Podoplanin-stained micro lymphatic vessels were observable all over a section, with tumor center having a trabs-like distribution of lymphatic vessels and with visible cancer embolus presented in part of vessels. Sections with high ANRIL expression had a significantly higher LMVD than those with low ANRIL expression (positive vs. negative: 11.36 ± 3.34 vs. 8.22 ± 2.31, t = 0.36, *P* < 0.01). Spearman correlation analysis showed that ANRIL expression positively correlated with LMVD (r = 0.66, *P* < 0.01).

**Figure 3:** ANRIL expression positively relates to lymphangiogenesis-related factors and LMVD in surgical specimens **A.** VEGF-C expression detected by immunohistochemistry; **B.** VEGFR-3 expression detected by immunohistochemistry; **C.** LYVE-1 expression detected by immunohistochemistry; **D.** Distribution of micro lymphatic vessels stained with CD34/Podoplanin, with CD34-stained vessels in bluish violet and Podoplanin-stained in bright red and presence of cancer embolus in some vessels. Note: ANRIL, antisense non-coding RNA in the INK4 locus; LMVD, lymphatic microvessel density.

**Table 3:** Spearman correlation analyses on the correlation between ANRIL expression and VEGF-C, VEGFR-3 and LYVE-1 in colorectal cancer

		ANRIL expression		χ^2^	*P*
		Low	High		
VEGF-C expression	-	10	7	14.14	0
	+	2	8		
	++	2	18		
	+++	12	49		
VEGFR-3 expression	-	17	29	13.31	0
	+	3	8		
	++	5	11		
	+++	1	34		
LYVE-1 expression	-	25	40	18.63	0
	+	0	6		
	++	1	19		
	+++	0	17		

Note: ANRIL, antisense non-coding RNA in the INK4 locus; ANRIL expression higher than the mean expression level is defined as high and otherwise low; The protein expressions of VEGF-C, VEGFR-3 and LYVE-1 are leveled as negative (−, 0 point), weakly positive (+, 1~2 points), positive (++, 3~4 points) and strongly positive (+++, ≥ 5 points).

### ANRIL expression in the colorectal cancer cell line

The results of TR-PCR and Northern blotting showed that SW480, HT29, LoVo and HCT116 had significantly higher ANRIL expression than HCoEpiC (all *P* < 0.05), with LoVo and HCT116 presenting strongest expression (Figure 4). In this context, we chose LoVo and HCT116 as the study subjects for our cell experiment.

**Figure 4:** ANRIL expressions in HCoEpiC, SW480, HT29, LoVo and HCT116 cell lines **A.** ANRIL mRNA detected by RT-qPCR; **B–C.** ANRIL expression detected by Northern blot. Note: ANRIL, antisense non-coding RNA in the INK4 locus; RT-qPCR, real-time fluorescent quantitative polymerase chain reaction; *** refers to *P* < 0.001 in comparison with ANRIL expression in HCoEpiC cell line.

### Influence of ANRIL expression in cell migration and cell invasion

The width of the scratch was observed under an inverted optical microscope at 0 hour and 24 hour after scratching assay (Figure 5). LoVo cells presented a relative migration distance of 0.95 ± 0.08 mm in blank group, 0.86 ± 0.11 mm in si-NC group and 0.51 ± 0.02 mm in si-ANRIL group and HCT116 cells had a relative migration distance of 0.62 ± 0.13 mm in blank group, 0.71 ± 0.09 mm in si-NC group and 0.33 ± 0.03 mm in si-ANRIL group. Statistically, the relative migration distance was significantly shorter in si-ANRIL group when compared with blank group and si-NC group (both *P* < 0.05). Blank group and si-NC group showed no significant difference in their relative migration distances (*P* > 0.05). Besides, si-ANRIL group had smaller numbers (29 ± 2LoVo cells and 42 ± 11 HTC116 cells) of invasive cancer cells than blank group (89 ± 13 LoVo cells; 92 ± 16 HTC116 cells) and si-NC group (90 ± 11 LoVo cells; 89 ± 18 HTC116 cells) (all *P* < 0.05) while no significant difference was identified between blank group and si-NC group (all *P* > 0.05) (Figure 6).

**Figure 5:** In-vitro cell mobility of cancer cell lines detected by scratch assay after transfection with siRNA for ANRIL **A.** The width of the scratch observed with LoVo cell line under an inverted optical microscope at 0 hour and 24 hour after scratching assay; **B.** Statistical comparisons of the width of the scratch observed with LoVo cell line among si-RNA group, si-NC group and blank group. **C.** The width of the scratch observed with HCT116 cell line under an inverted optical microscope at 0 hour and 24 hour after scratching assay; **D.** Statistical comparisons of the width of the scratch observed with HCT116 cell line among si-RNA group, si-NC group and blank group. Note: ANRIL, antisense non-coding RNA in the INK4 locus; siRNA, small interfering RNA; NC, negative control.

**Figure 6:** In-vitro invasion activity of LoVo cell line and HCT116 cell line detected by Transwell invasion assay after transfection with siRNA for ANRIL in si-ANRIL group, si-NC group and blank group Note: ANRIL, antisense non-coding RNA in the INK4 locus; siRNA, small interfering RNA; NC, negative control; * refers to *P* < 0.05 in comparison with blank group; ** refers to *P* < 0.01 in comparison with blank group; ^#^ refers to *P* < 0.05 in comparison with si-NC group; ^##^ refers to *P* < 0.01 in comparison with si-NC group.

### Influence of ANRIL expression on the in vitro lymphangiogenesis and lymphatic migration

HLECs were cultured with TSNs. The result of tube-formation and Transwell migration revealed that si-ANRIL group had a smaller number of tube junction (Figure 7) and migrated HLECs in comparison with blank group and si-NC group (Figure 8) (all *P* < 0.05). No significant difference was found between blank group and si-NC group in their number of tube junction or migrated cell (*P* > 0.05).

**Figure 7:** In-vitro ability of TNS-cultured HLECs in tube-formation after transfection with siRNA for ANRIL in si-RNA group, si-NC group and blank group Note: TNS, tumor culture supernatants; HLEC, human lymphatic endothelial cell; ANRIL, antisense non-coding RNA in the INK4 locus; siRNA, small interfering RNA; NC, negative control; ** refers to *P* < 0.01 in comparison with blank group; ^##^refers to *P* < 0.01 in comparison with si-NC group.

**Figure 8:** In-vitro cell migration of TNS-cultured HLECs detected by Transwell migration assay after transfection with siRNA for ANRIL in si-ANRIL group, si-NC group and blank group Note: TNS, tumor culture supernatants; HLEC, human lymphatic endothelial cell; ANRIL, antisense non-coding RNA in the INK4 locus; siRNA, small interfering RNA; NC, negative control; ** refers to *P* < 0.01 in comparison with blank group; ^##^ refers to *P* < 0.01 in comparison with si-NC group.

### Influence of ANRIL expression on the lymphangiogenesis-related factors in the colorectal cancer cells

mRNA and protein expressions of VEGF-C, VEGFR-3 and LYVE-1 in the colorectal cancer cells were measured by RT-PCR and Western Blotting (Figure 9–10). After the downregulation of ANRIL in those cells, a decrease in the expressions of VEGF-C, VEGFR-3 and LYVE-1 was observed in all three groups, with si-ANRIL group presenting significantly lower expressions of VEGF-C, VEGFR-3 and LYVE-1 than both blank group and si-NC group (all *P* < 0.05). However, no significant difference was observed between blank group and si-NC group in the expressions of VEGF-C, VEGFR-3 and LYVE-1 (all *P* > 0.05).

**Figure 9:** mRNA expressions of VEFG-C, VEFGR-3 and LYVE-1 detected by RT-qPCR in LoVo and HTC116 cell lines after transfection with siRNA for ANRIL in si-ANRIL group, si-NC group and blank group Note: ANRIL, antisense non-coding RNA in the INK4 locus; siRNA, small interfering RNA; NC, negative control; RT-qPCR, real-time fluorescent quantitative polymerase chain reaction; * refers to *P* < 0.05 in comparison with blank group;** refers to *P* < 0.01 in comparison with blank group; ^#^ refers to *P* < 0.05 in comparison with si-NC group;^##^ refers to *P* < 0.01 in comparison with si-NC group; ^###^ refers to *P* < 0.001 in comparison with si-NC group.

**Figure 10:** Protein expressions of VEFG-C, VEFGR-3 and LYVE-1 detected by Western blot in LoVo and HTC116 cell lines after transfection with siRNA for ANRIL in si-ANRIL group, si-NC group and blank group Note: ANRIL, antisense non-coding RNA in the INK4 locus; siRNA, small interfering RNA; NC, negative control; * refers to *P* < 0.05 in comparison with blank group; ** refers to *P* < 0.01 in comparison with blank group; *** refers to *P* < 0.001 in comparison with blank group; ^#^refers to *P* < 0.05 in comparison with si-NC group;^##^refers to *P* < 0.01 in comparison with si-NC group.

### Influence of ANRIL expression on tumor growth in the mouse model of colorectal cancer

All the included mice lived through the whole experiment and tumor formation rate was 100%. At 3~4 days after hypodermic inoculation, growing tumor nodules (tumor size of 4-6 mm) were observed (Figure 11A). As shown in the tumor growth rate curves of sh-NC group and sh-ANRIL group (Figure 11D), sh-ABRIL group presented a significant lower growth rate than sh-NC group (*P* < 0.05). This experiment ended on the 28^th^ day, with gross tumor volume as 1018.15 ± 59.12 mm^3^ in sh-ANRIL group and as 2794.53 ± 75.63 mm^3^ in sh-NC group. By statistical analysis, the difference between sh-ANRIL group and sh-NC in the gross tumor volume was significant (*P* < 0.05). For observation, general tumor samples were collected from both sh-NC group and sh-ANRIL group. sh-NC group had tumors rich in blood supply, crispy in texture, closely embedded into rat's skin, difficult to peel from the skin and easy to bleed when peeling and also they presented infiltration in the surrounding skin and subcutaneous tissue and anabrosis on mice' skin (Figure 11B). However, tumors in sh-ANRIL group were easy to peel and had slight infiltration in surrounding tissues (Figure 11C). Pathological sections were made out of tumors for observation. Sections from sh-NC group presented loose cell arrangements and massive necrosis of tumor cells while those from sh-ANRIL group exhibited dense cell arrangements and a large number of blood cells (Figure 11E).

**Figure 11:** A mouse model of orthotopically transplanted colon tumor **A.** tumor transplantation is successful in all the included mice after transfection with sh-ANRIL; **B.** Transplantation tumors collected from sh-ANRIL group; **C.** Transplantation tumors collected from sh-NC group; **D.** Tumor growth rates of sh-ANRIL group and sh-NC group from the 5^th^ day to the 28^th^ day. **E.** Presentation of stained sections HE staining; sections were made out of tumors tissues from sh-ANRIL group and sh-NC group. Note: sh-ANRIL, short hairpin RNA for ANRIL; NC, negative control; *** in D refers to *P* < 0.001 in comparison with sh-ANRIL group.

### Influence of ANRIL expression in lymphatic metastasis and lymphangiogenesis in the mouse model of colorectal cancer

Anti-pan-cytokeratin was used to detect lymphatic metastasis in the naked mice with immunohistochemistry. Sections with lymphatic metastasis presented tumor cells in brown (Figure 12A) while sections without lymphatic metastasis only had tumor cells in blue (Figure 12B). Lymphatic metastasis rate was 100% (10/10) in sh-NC group (10 mice were positively-stained with anti-pan-cytokeratin) and 20% (2/10) in sh-ANRIL group. Frequency of transferred lymph nodes was 4.06 ± 2.47 node/mouse in sh-NC and 1.02 ± 0.17 node/mouse in sh-ANRIL group. Apparently, sh-ANRIL group had a significantly lower number of transferred lymph node than sh-NC group (*t* = 2.746, *P* = 0.025). These transplanted tumors received dehydration, fixation and slicing for immunohistochemistry (Figure 13). We found that sh-ANRIL group had smaller LMVD than sh-NC group (sh-ANRIL vs. sh-NC: 2.31 ± 1.38 vs. 7.14 ± 3.00; *t* = 3.27, *P* = 0.01).

**Figure 12:** Lymph node metastasis in the mice with transplanted colon tumor detected with immunohistochemistry and CK antibody after transfection with sh-ANRIL **A.** In mice with lymphatic metastasis, CK was positive and tumor cells were stained with immunohistochemistry as dark brown; **B.** In mice without lymphatic metastasis, CK was negative; lymphatic cells presented in blue and no cells were stained with immunohistochemistry as dark brown; Note: sh-ANRIL, short hairpin RNA for ANRIL; CK antibody, anti-pan-cytokeratin.

**Figure 13:** Stained lymphatic vessels of the transplantation tumors in the included mice with immunohistochemistry

### Expressions of VEGF-C, VEGFR-3 and LYVE-1 in the transplanted tumors

Following dehydration, fixation and slicing, these tumors got immunohistochemistry. After immunohistochemistry, protein staining of VEGF-C, VEGFR-3 and LYVE-1 was significantly slighter in sh-ANRIL group than in sh-NC group (Figure 14). Besides, total proteins were extracted from transplanted tumors for Western blotting assay. The results of protein detection demonstrated that sh-ANRIL group had lower expressions of VEGF-C, VEGFR-3 and LYVE-1 than sh-NC group (all *P* < 0.05) (Figure 15).

**Figure 14:** After dehydration, fixation and slicing, the transplanted tumors form both sh-ANRIL group and sh-NC group were stained with immunohistochemistry for the detecting the expressions of ANRIL, VEFG-C, VEFGR-3 and LYVE-1 Note: sh-ANRIL, short hairpin RNA for ANRIL; NC, negative control.

**Figure 15:** Expressions of ANRIL, VEFG-C, VEFGR-3 and LYVE-1 detected by Northern blot in the transplanted tumors from both sh-ANRIL group and sh-NC group **A.** Electrophoretogram presenting the expressions of VEFG-C, VEFGR-3 and LYVE-1 in sh-ANRIL group and sh-NC group; **B.** Statistical analyses on the expressions of VEFG-C, VEFGR-3 and LYVE-1 in sh-ANRIL group and sh-NC group. Note: ANRIL, antisense non-coding RNA in the INK4 locus; sh-ANRIL, short hairpin RNA for ANRIL; NC, negative control; *** refers to *P* < 0.001 in comparison with sh-NC group.

## DISCUSSION

In our study, we observed significantly overexpressed ANRIL mRNA in patients with colorectal cancer and a close association between ANRIL expression and the clinicopathologic features of colorectal cancer. Concordantly, Lin *et al*. also identified increased ANRIL expression. remarkably associated with clinicpathologic features of colorectal cancer [16]. In agreement with previous studies [16, 25], we found that up-regulated ANRIL expression may be a risk factor for poor prognosis of colorectal cancer along with lymph node metastasis and distant metastasis.

Interestingly, we also found that patients with high ANRIL expression also presented higher expressions of VEFG-C, VEGFR-3 and LYVE-1. LYVE-1 is a key specific marker for lymphatic endothelial cell (LEC), responsible for transporting hyaluronan (HA) on the LEC surface [26]. By the binding of HA to LYVE-1, lymphangiogenesis is started [27]. VEGF-C is a major modulator in the postnatal development of lymphangiogenesis; its binding to VEGFR-3 is a mature marker for lymphangiogenesis [28, 29]. Previous study suggested that increased LYVE-1 and overexpressed VEFG-C work together to form lymphatic vessel [30, 31]. Consistently, our study also found higher LMVD in patients with higher ANRIL expression, that is, patients with higher VEFG-C, VEGFR-3 and LYVE-1. Besides, using Spearman correlation analyses, we observed a positive correlation between ANRIL expression and the expression of VEFG-C, VEFGR-3 and LYVE-1. Taken together, we believe that increased ANRIL may act as a driver for lymphangiogenesis via the upregulation of LYVE-1, VEFG-C and VEGFR-3 and therefore lead to lymphatic metastasis.

In vitro cell experiments, we found that ANRIL suppression apparently reduced activity in their invasion and migration. Qiu et al. also suggested that down-regulation of ANRIL leads to lowered activity in SOC (for serious ovarian cancer) cell migration and invasion [32]. In addition, down-regulated ANRIL could repress in-vitro lymphangiogenesis and migration of endothelial cells, accompanied with reduced expression of LYVE-1, VEFG-C and VEGFR-3. Chen et al. suggested that inhibition of ANRIL could increase the transforming growth factor β1 [24]. While Cui et al. reported that transforming growth factorβ1 in human lung fibroblasts could downregulate the expression VEFG-D which is also an important factor in lymphangiogenesis [33, 34]. These results implied that downregulation of ANRIL expression may be an effective way to control metastasis through inhibiting lymphangiogenesis in the colorectal cancer.

In the mouse model, we observed that mice with down-regulated ANRIL had significantly lowered tumor growth rates, suggesting that downregulation of ANRIL may inhibit the growth of tumor cell. As suggested by Zhang et al., ANRIL has a facilitating role in tumor growth [35]. Inevitably, downregulated ANRIL may lead to suppressed tumor growth. We observed that, tumors in mice with down-regulated ANRIL presented considerable cell death. ANRIL has a direct role in binding polycomb group proteins to *INK4a* and *INK4b* loci to repress gene expression of *p16^INK4a^*, p14ARF** and *p15^INK4b^* [36]. p16^INK4a^ and p15^INK4b^ are well-accepted inhibitor of the cyclin-dependent kinase 4 while p14ARF is responsible for stabilizing p53 through interaction with murine double minutesute 1 [37]. By suppressing or activating *p16^INK4a^*, p14ARF** and *p15^INK4b^*, ANRIL could accelerate the cell cycle of tumor cells. Several studies have reported that increased ANRIL could promote cell proliferation and inhibits cell apoptosis [38, 39]. We also found that downregulation of ANRIL in mouse model lead to repressed lymphangiogenesis, lymphatic metastasis, and decreased expressions of LYVE-1, VEFG-C and VEGFR-3. These results suggested that ANRIL expression may be a prognostic and therapeutic factor for colorectal cancer via its role in lymphangiogenesis and lymphatic metastasis.

In conclusion, our study provides solid evidence that ANRIL is over expressed in colorectal cancer. Through downregulation of the overexpressed ANRIL in colorectal cancer, expressions of LYVE-1, VEFG-C and VEGFR-3, lymphangiogenesis and lymphatic metastasis could be repressed. Therefore, ANRIL may be a useful prognostic and therapeutic factor for colorectal cancer. For validating of the effect of ANRIL on the development of colorectal cancer, we need to make more efforts to figure out the pathways ANRIL relates to lymphangiogenesis and lymphatic metastasis.

## MATERIALS AND METHODS

### Ethic statement

This research was carried out in strict consistence with the protocols established by the Ethics Committee of Central South University. All the experimental procedures in this study were in accordance with the Declaration of Helsinki [20]. The informed consents were obtained from all subjects participated in this study or their families and this study was approved by the local institutional review board.

### Source of specimens

In our study, we enrolled 108 patients with colorectal cancer who hospitalized in The Third Xiangya Hospital of Central South University between November 2008 and November 2010. Surgical specimens and paired normal colorectal mucosae (≥ 8 cm away from the paracarcinoma) were collected from the enrolled patients during excisions. All the patients were pathologically diagnosed with colorectal cancer and free of chemotherapy or radiotherapy before excision and also had complete clinical and pathological data. Among 108 patients, 59 were male and 49 female, 47 were at age of ≤ 50 and 61 of > 50 (mean age of 49.78 ± 16.08), 61 had colon tumors and 47 had rectal tumor, 54 presented a tumor of size ≤ 5 cm and 54 of size > 5 cm (mean tumor size of 6.76 ± 4.06 cm), 23 carried poorly-differentiated tumors and 85 moderately and highly-differentiated tumors by tumor histology, 50 exhibited lymphatic metastasis and 58 no lymphatic metastasis, 20 had distant metastasis and 88 no distant metastasis, 59 were at stage I + II and 49 at stage III + IV by Tumor-Node-Metastasis staging prescribed by Union for International Cancer Control and American Joint Committee On Cancer in 2003 [21], 74 had tumors invading plasma membrane and 34 had tumors plasma membrane invasion-free and 56 were at stage A+B and 52 at C+D by Dukes staging [21] (Table 1).

### Follow-up

Our follow-up was conducted through phone contacts and medical recordings, altogether lasting for 5 years from the discharge after systematic treatment to November 2015. If patients were still alive at the end of the follow-up, the follow-up data was censored at the latest contact. For patients lost to follow up, the last data census applied. Among 108 follow-ups, 102 were followed up until the end and 6 were lost. Survival time was calculated by the month. Overall survival (OS) was defined as the duration from the excision to death caused by any reason.

### Cell culture

Four colorectal tumor cell lines, HT29, SW480, HCT116 and LoVo, were purchased from Shanghai Institute of Cell Biology, Chinese Academy of Sciences. These cell lines were incubated with 10% fetal bovine serum (FBS), penicillin (100U/ml), streptomycin (100μg/ml) and glutamine RPMI1640 solution (2mmol/L; Hyclone Company, Logan, USA) at 37°C under 5% CO_2_. Normal colonic epithelial cell line, HCoEpic (Sciencell Research Laboratories, Carlsbad, USA), was cultured in DMEM solution at 37°C under 5% CO_2_. Human lymphatic endothelial cells (HLECs; Sciencell Research Laboratories, Carlsbad, USA) were cultured in endothelial cell medium (ECM; ScienCell Research Laboratories, Carlsbad, USA) with 5% FBS and endothelial growth medium supplements (VEGF-C-free) [22].

### Cell grouping and transfection

At 24 hours before transfection, cells at logarithmic phase were digested with trypsin and counted and the cell concentration was adjusted to 2×10^5^ cells/ml. Cell suspension (200 μl) was seeded on a 6-well plate containing 2 ml DNEM solution (antibiotic-free; 10% FBS). For this experiment, HCT116 and LoVo cells were divided into three groups: si-ANRIL group transfected with small interfering RNA (siRNA) for ANRIL; si-NC group transfected with negative control siRNA; Blank group without transfection. After all the cells reached a confluence of 50%-60%, transfection was conducted according to the instructions of Lipofectamin^TM^ 2000 (Invitrogen, Carlsbad, USA) and the sequence of si-ANRIL, GGUCAUCUCAUUGCUCUAU, was purchased from Shanghai GenePharma Co., Ltd [23]. After 48 hours, we harvested tumor culture supernatants (TSNs) and had them centrifuged and preserved in aliquots at −80°C. The transfected cell lines were screened for stable expressions of si-ANRIL by applying puromycin in the culture medium for 10 days.

### A mouse model of orthotopically transplanted colon tumor

LoVo cells were seeded in a 6-well plate at a confluence of 60% and then were transfected with short hairpin RNA (shRNA) for ANRIL (sh-ANRIL) and negative control shRNA (sh-NC). Sh-ANRIL was synthesized by Genechem (Shanghai, China) and its sequence was GGTCATCTCATTGCTCTATCC [23]. Then sh-ANRIL and sh-NC LoVo cells continued to be cultured in G418 (200 μg/ml) and then selected with full-dose G418 (300 μg/ml) at two weeks before inoculated to mice. For the inoculation, anchorage-dependent cells at logarithmic phase were gathered and then digested with 0.25% trypsin, followed by centrifugation, recovery and resuspension in serum-free DMEM. Subsequently, the cultured cells were re-centrifuged at 1000 rpm and room temperature for 5 minutes and again re-suspended in serum-free DMEM after the supernatant was removed. These cells were inoculated to ten naked mice which were equally allocated into sh-ANRIL and sh-NC group, sh-ANRIL group carrying sh-ANRIL LoVo cells while sh-NC group with sh-NC LoVo cells. After the inoculation, the mice were put under close observation of their systematic condition and weight, their movement condition, the growth rate and the volume of the implantation tumor. The volume of the implantation tumor was calculated as the value of l/2 × ab^2^, with a referring to the major axis and b to the minor axis. The length measurement was conducted with a vernier caliper and a tumor growth curve was drawn. At 28 days after the inoculation, the mice were killed by vertebral dislocation, and then the tumors in them were cut off and exploration in their pleuroperitoneal cavity was performed. Collected mouse tumors were fixed in 10% formaldehyde, followed by dehydration, paraffin embedding, slicing and hematoxylin-eosin (HE) staining. Besides, Immunohistochemistry assays were conducted to develop CK, ANRIL, VEFGF-C, VEDFR-3 and LYVE-1 and the lymph vessel density was observed under light microscope after dyeing.

### Real-time fluorescent quantitative polymerase chain reaction (RT-qPCR) for detecting mRNA expression

The whole RNA was extracted using Trizol. An ultraviolet spectrometry photometer was used to detect its purification and concentration and agarose gel electrophoresis was conducted for detecting the integrity of RNA. For reverse transcription, a Primescript^TM^ RT reagent Kit (TaKaRa; Dalian, Liaoning, China) applied. The Stratagene Mx3000P^TM^ Real Time PCR System (Agilent Technologies; Santa Clara, California, USA) with SYBR® Premix Ex Taq^TM^ (TaKaRa) reagent was: one cycle at 95°C for 30 s, 40 cycles at 95°C for 5 s, and one cycle at 60°C for 20 s. The sequences of amplimers: for ANRIL-1, the forward was 5′-TCACTGTTAGGTGTGCTGGAAT-3′ and the reverse was 5′-CCTCTGATGGTTTCTTTGGAGT-3′; for ANRIL-2, the forward was 5′- CCGCTCCCCTATT CCCCTTA-3′ and the reverse is 5′- CCTGATTGGCGGA TAGAGCA-3′; for GAPDH, the forward was 5′- TCAACG GATTTGGTCGTATTG-3′ and the reverse was 5′- TGGGTGGAATCATATTGGAAC-3′. ANRIL-1 primers were applied for amplification in colon tumor tissue while ANRIL-2 primers designed for use in cell [24], and GAPDH acted as the internal reference. For VEGF-C, the forward was 5′- GCCCCAAACCAGTAACAATC-3′ and the Reverse was 5′-GTTGAGTCATCTCCAGCATCC-3′, for VEGFR-3, the forward was 5′-AGCCATTCATCAA CAAGCCT-3′ and the reverse was 5′-GGCAACAGCT GGATGTCATA-3′ and for LYVE-1, the forward was 5′-ATCCCATATTCAACACTCAA′ and the reverse was 5′-CCTTTACTACTTTGGTTTCG-3′. The results of PCR were analyzed with Opticon-Monitor 3 software (Bio-Rad Laboratories, California, USA). The threshold was manually set as the lowest point where logarithmic amplification curves started to raise in parallel and the threshold cycle was recorded accordingly. The expression of ANRIL was calculated with 2^−ΔΔCt^ method and all the experiments were conducted in triplicate.

### Northern blot

Total RNA (20 ug) was extracted for electrophoresis on gel containing formaldehyde. After electrophoresis, RNA was transferred into Hybond-N + nylon membrane (Amersham), followed by fixation with ultraviolet crosslinking, pre-hybridization (68°C, 30 minutes) and probe labeling. A random primer labeling kit (Prime-a-Gene, Promega) was used for ANRIL probe labeling and probe (25 ng) was labeled with [α-32P] DCTP (3000 CI/mmol). Afterward, the membrane was cultured in hybridization solution (68°C, overnight) along with the probe. Subsequently, the membrane was washed with 1×SSC/0.1% SDS at 68°C (15 minutes; twice) and then radiographed at −70°C. ANRIL expression was expressed as ratio between the grey value and that of β-actin.

### Western blot

After the extraction of total protein with lysis buffer, the protein concentration was measured by Bicinchoninic acid (BCA) assay. Later, the extracted protein (50 μg) got electrophoresis under constant voltage in 10% sodium dodecyl sulfate-polyacrylamide gels (SDS-PAG), followed by wet-transfer into a polyvinylidene fluoride (PVDF) membrane. The transferred membrane was blocked with 5% skim milk powder at room temperature, followed by the addition of primary antibodies (VEGF-C: ab135506, 1:500, Abcam, Cambridge, UK; VEGFR-3: ab51874, 1:800, Abcam, Cambridge, UK; LYVE-1: ab33682, Abcam, 1:100, Cambridge, UK). Then this sample was incubated overnight at 4°C on a shaking table and washed for 3 times, after which goat-anti-rabbit horseradish peroxidase conjugated antibodies were added (ab6721, Abcam, 1:2000, Cambridge, UK) as secondary antibodies. Subsequently, the sample was incubated at room temperature for 1 hour, followed by coloration with enhanced chemiluminescence (ECL) plus reagent and imaging. The calculation of the grey level of target bands was conducted with Synegene gel imaging system and GeneTools was employed for analyses on protein bands. β-actin was used as internal reference (ab194952, 1:1000, Abcam, Cambridge, UK) for adjustment.

### Immunohistochemical staining

After being dewaxed, the paraffin sections were immersed in 3% H_2_O_2_ methanol for digestion of endogenous peroxidase and then in 0.5% bovine serum albumin for blockage of non-specific antibodies. After that, sections were incubated with primary antibodies (VEGF-C: ab135506, Abcam, Cambridge, UK; VEGFR-3: a51874, Abcam, Cambridge, UK; LYVE-1: ab33682, Abcam, Cambridge, UK) in a wet box at 4°C overnight. Subsequently, the biotin labeling secondary antibodies were added (ab6721, 1:2000, Abcam, Cambridge, UK) and then streptavidin-horseradish peroxidase (Zhongshanjinqiao Biotechnology Inc., Bejing, China) was also added. After that, DAB coloration, hematoxylin staining, regular dehydration and hyalinization and blockage were conducted. For double-labeling immunohistochemistry, Podoplanin and CD34 were added to the sections, followed by incubation with primary antibodies (4°C, overnight). Then the sections received PBS rinse (3 times × 3 minutes). Subsequently, the secondary antibodies (15 minutes, 37°C) were added to the sections. Then they received incubation with streptavidin–alkaline phosphatase conjugates (37°C, 15 minutes) and coloration with BCIP/NBT solution for coloration. Later, the sections got 15-minute incubation with double-staining enhancer at 37°C. After the first 15-minute serum blocking, the sections were cultured with a second primary antibody and then blocked with serum again Next, biotin-labeled secondary antibody was added to the sections for 15-minute incubation at 37°C, followed by incubation with streptavidin–alkaline phosphatase conjugates for 15 minutes at 37°C. After that, AEC solution was added to the sections for coloration and a micro scope was used to observe and record the color of the sections. Then hematoxylin was added to the sections for re-dyeing. Through the experiment, sections all received PBS rinse three times before entering the next step. In the end, the sections were washed with running water and then dehydrated, transparentized and sealed with glycerinum.

### Result interpretation of immunohistochemistry

Ten high-power fields were selected in random for observation (100 cells/field). Successfully-stained proteins of ANRIL, VEGF-C, VEGFR-3 and LYVE-1 were clearly localized in the cytoplasm as granules, from light yellow to dark brown By the staining intensity, protein expressions scored 0 point (colorless), 1 point (light yellow), 2 points (brownish yellow) and 3 points (dark brown); while by rates of positive cell, protein expressions were marked as 0 point (≤ 10%), 1 point (10%~25%), 2 points (25%~50%), and 3 points (> 50%). In the double-labeling immunohistochemistry, Podoplanin and CD34 were differentially expressed in micro lymph vessels and capillaries, while the former was in bright red and the latter in dark violet. Lymph vessels had endotheliocytes stained as bright red (positive Podoplanin expression), monolayer endothelial cells-constructed tube but had no basement membrane and smooth muscle cell in the periphery and no blood cells in the tube. Those vessels which exhibited in bright red but with no tube structure were not considered as lymph vessel. Subsequently, we selected vessel-rich regions in the sections at low magnification (× 100). Afterward, three fields of the vessel-rich regions were randomly selected for counting of lymphatic microvessel density (LMVD) at ×200 magnifications. The final LMVD was defined as the average of the value observed from the three fields.

### Scratch assay for cell migration in vitro

LoVo and HCT116 single cell suspensions (2 ml for each) were seeded into 6-well plates at a density of 1 × 10^5^ cell/ml. For each group, three repeated holes were set in parallel. Then LoVo cell and HCT116 cell were transfected with si-NC and si-ANRIL using the method as used before. AT 16 hour after the transfection, the injectable transfection suspension was abandoned. After that, the cells continue to be cultured with complete culture solution for another 12 hours. A sterile micro pipette tip was used to vertically scratch in the 6-well plates. After scratching, the cells were washed with PBS buffer for twice and then incubated in serum-free solution. At 0 hour and 24 hour after incubation, the width of the scratch was measured and compared among groups under an inverted fluorescence microscope (IX-71). For the measurement and comparison, 5 fields (×100) were randomly selected for each group and then photographed.

### Invasion assay

Two 24-well plates and BD Falcon cell culture inserts with 8.0-μm pores (BD Biosciences, Franklin Lakes, NJ, USA) were used for cell culture. The bottom of the inserts was pre-coated with Matrigel (BD Biosciences). In the lower chamber of the 24-well plate, 600 μl 10% FBS/DMEM was placed while in the upper chamber were LoVo and HCT116 cells. Cells were incubated at 37°C for 24 hours. After incubation, we collected cells that invaded the membrane, followed by fixation in 1% paraformaldehyde, staining with crystal violet and cell counting under an optical microscope (× 200). Three fields were selected in random for cell counting.

### Migration assay

Two Transwell chambers (BD Biosciences) was used for migration assay. The upper chamber contained serum-free medium and HLECs (2 × 10^4^) while the lower chambers carried the TSNs derived from LoVo and HCT116. After 10-hour incubation, HLECs that migrated to the lower membrane surface were fixed, stained and counted as done in the invasion assay.

### Tube formation Assay

Tube formation assay was conducted with a 48-well plate containing Matrigel (75μl/well) and serum-free ECM (75μl/well). Then, HLECs (2 × 10^4^) were incubated in ECM (100 μl) and TSNs (400 μl) on the Matrigel layer in each well. After 4 hours, tube formation was observed using phase-contrast microscopy (× 40) and photographed [22].

### Statistical analyses

Data analyses were conducted using SPSS 19.0 (SPSS Inc., Chicago, IL, USA). Numerical data expressed as mean ± standard deviation ($\bar{x}\pm \text{s}$) and put to normality test. Comparisons between two groups of numerical data were conducted by t test and those among more than two groups were performed with One-way analysis of variance (a homogeneity test for variance was needed before analyses). Pairwise comparisons between means were conducted with least significant difference test. Categorical data were expressed with frequency or percentage and comparisons were conducted by Chi-square test. Survival rate was calculated with Kaplan-Meier method and prognostic factors were screened with Cox regression model. *P* < 0.05 indicated significantly statistical difference.
